The article "Primary Chondrosarcoma of the Right Fourth Rib Resected at the Marginal Margin: A Case Report" was published in 2023. Journal: Cureus.

# Primary Chondrosarcoma of the Right Fourth Rib Resected at the Marginal Margin: A Case Report

**DOI:** 10.7759/cureus.51251

**Published:** 2023-12-28

**Authors:** Ryusei Yoshino, Masaki Nakatsubo, Nanami Ujiie, Nana Yoshida, Sayaka Yuzawa, Masahiro Kitada

**Affiliations:** 1 Thoracic Surgery and Breast Surgery, Asahikawa Medical University Hospital, Asahikawa, JPN; 2 Diagnostic Pathology, Asahikawa Medical University Hospital, Asahikawa, JPN

**Keywords:** marginal margin, surgery, thoracic surgery, ribs, chondrosarcoma

## Abstract

Primary chondrosarcoma of the ribs is relatively rare, and its basic treatment is surgical resection. In cases with positive resection margins, additional resection is considered, but its indications are unclear. However, reported cases with positive resection margins have been limited. We report a 71-year-old man whose medical checkup revealed an abnormal shadow in the chest. The findings from chest computed tomography, axial T2-weighted magnetic resonance imaging (MRI), and contrast-enhanced MRI led to a diagnosis of chondrosarcoma of the right fourth rib, and surgical resection was performed. The chest wall defect was reconstructed with a Marlex mesh. Postoperative histopathologic diagnosis was grade 2 chondrosarcoma. Gross resection margins, which were marginal, were negative, and the resection margin was grade 1. The patient was followed up without adjuvant therapy and did not undergo additional surgery. For chondrosarcomas with negative gross margins but a marginal margin, additional resection should be considered depending on the histologic grade of the margins. In cases with extensive resection of the chest wall, it is useful to reconstruct the chest wall while paying careful attention to infection control.

## Introduction

Chondrosarcoma is included in the category of chondrogenic tumors, is designated as sarcoma arising from the cartilage matrix, and is associated with local destruction or metastasis [1]. Chondrosarcoma commonly develops in the pelvis and long bones, whereas primary chondrosarcoma of the ribs is a relatively rare disease [1,2]. The differential diagnoses included benign enchondroma. Because chondrosarcoma may exhibit atypical presentation, differentiation may be difficult [3]. In consideration of the clinical features of enchondroma, including the peak age of onset of 10-39 years and rare incidence on the trunk (including the pelvis and ribs), differentiation is often performed before surgery [1].

The basic treatment is surgical resection, and a complete cure cannot be expected with chemotherapy or radiotherapy [4]. Thus, complete surgical resection is one of the key treatment strategies. Consequently, reports of positive resection margins have been extremely limited. Although this case is that of an R1 resection, the patient's decision not to have additional resection gave us the opportunity to follow a positive resection margin of the right fourth rib. This case has not progressed to date. Since there are very few reports of a condition similar to that of our reported case, we consider this report to be of value. In addition, chest wall reconstruction was performed due to the wide resection. We report this case along with a literature review.

The article "Primary Chondrosarcoma of the Right Fourth Rib Resected at the Marginal Margin: A Case Report" was published in 2023. Journal: Cureus.

## Case presentation

The patient was a 71-year-old man. Although chest radiography performed during a medical checkup in 2019 revealed a mass shadow in the right ribs, he did not undergo a detailed examination. Approximately two years later, an abnormal shadow was detected in the right ribs again. Detailed examination with chest computed tomography (CT) revealed a mass in the right fourth rib. Based on a CT-guided biopsy performed on this site, chondrosarcoma (grade 1>2) was diagnosed. The patient was referred to our department for surgery. He had no remarkable medical history, including cardiac or respiratory diseases. His family history was unremarkable. He had smoked 10-15 cigarettes per day for 17 years (age: 17-34 years) and was a social drinker.

His height was 171 cm, weight was 77 kg, and body mass index was 26.3. The respiratory sound over the chest was clear, and mild tenderness was noted in the right precordial area on the fourth rib. A 40 × 45 mm bone-like hard well-circumscribed mass was palpated subcutaneously at the same site. The laboratory findings on admission were as follows. Hematologic test results, including complete blood cell count, lactate dehydrogenase, and alkaline phosphatase, were within the normal ranges. The respiratory function test and electrocardiography showed no abnormal findings. Chest radiography showed an abnormal shadow in the right middle lung field (Figure 1). Chest CT showed a 34 × 33 mm mass shadow with internal calcification in the right fourth rib (Figure 2). Chest magnetic resonance imaging (MRI) showed a 41 × 32 × 48 mm hyperintense mass in the right fourth rib on axial T2-weighted images. Contrast-enhanced MRI showed a heterogeneous enhancement predominantly in the periphery. There was no other evidence of distant metastasis on the thoracoabdominal CT scan. Therefore, an 18-fluoro-deoxyglucose positron emission tomography (FDG-PET) scan was not performed in this case.

**Figure 1:** Chest radiograph (frontal view) A tumor shadow with indistinct boundaries in the right middle lung field.

**Figure 2:** CT chest findings (mediastinal condition) A 34 mm x 33 mm large tumor shadow with internal calcification at the fourth rib.

The article "Primary Chondrosarcoma of the Right Fourth Rib Resected at the Marginal Margin: A Case Report" was published in 2023. Journal: Cureus.

The surgical findings were as follows. First, the incision method was determined by considering the possibility of obtaining an adequate resection margin at the site on the fourth rib where the tumor was thought to be located. A transverse incision was made across the pectoralis muscle from its lateral border to the right parasternal region (Figure 3a). A thoracoscope was used to identify the tumor, and markings were made to obtain a margin of at least 20 mm. The tumor was inspected and resected from the third to fifth ribs vertically and with a 20 mm margin in both horizontal directions. Therefore, the gross resection margins were determined to be negative. A thoracic drain was placed prior to the placement of the mesh for the reconstruction of the defect. The defect measured approximately 100 × 90 mm and was reconstructed with the Marlex mesh (Figure 3b). Specifically, we used 2-0 nylon sutures to suture and fixed the rib margins to the ribs and the intercostals to the surrounding tissues (such as the intercostal muscles).

**Figure 3:** Skin incision lines in the actual surgery (a) A transverse incision was made from the lateral border of the pectoralis major muscle to the right parasternal area. (b) After reconstruction with the mesh.

The examination of the resected sample showed a 5.8 × 3.5 × 4.3 cm tumor, with protruding growth mainly in the fourth rib (Figure 4). Histopathologically, the tumor proliferated in the cartilage matrix in a lobular manner and infiltrated into the surrounding soft tissues beyond the bone cortex. The chondrosarcoma was heterogeneous with components comprising approximately 80% grade 1 and 20% grade 2 disease (Figures 5a-5c), leading to the diagnosis of grade 2 primary chondrosarcoma of the rib. The tumor was removed grossly, but the grade 1 chondrosarcoma was exposed to the resection margin of the fourth rib microscopically (Figure 6); therefore, the tumor was determined to be R1 resection, and the so-called resection margin was the marginal margin.

**Figure 4:** Findings of the resected specimen The tumor was resected as a single lump, including the chest wall and skin. The resection extended from the superior margin of the third rib on the cephalic side, the inferior margin of the fifth rib on the caudal side, the costal cartilage on the medial side, and a 3 cm resection margin from the tumor on the lateral side.

**Figure 5:** Histopathological findings of the tumor (a) The tumor is composed of grade 1 (left) and grade 2 (right) chondrosarcoma (HE stain, ×10) (b). Grade 1 chondrosarcoma shows a sparse proliferation of chondrocytes in the cartilage matrix (HE stain, ×40) (c). Grade 2 chondrosarcoma shows a relatively dense proliferation of chondrocytes with increased pleomorphism and myxomatous changes (HE stain, ×40).

The article "Primary Chondrosarcoma of the Right Fourth Rib Resected at the Marginal Margin: A Case Report" was published in 2023. Journal: Cureus.

**Figure 6:** Histopathological findings of the resected margin of the fourth rib A grade 1 chondrosarcoma is exposed to the resection margin (HE stain, ×10).

Furthermore, for the marginal margin, the patient was offered an additional resection, including a partial sternal resection, since this was a case of R1 resection. However, the patient did not strongly request surgery; thus, it was not performed. After a discussion with him, postoperative adjuvant therapy was not administered, either. While he has been carefully followed up every three months for approximately two years after surgery, he is still under observation without recurrence at present.

Written informed consent was obtained from the patient for this publication.

## Discussion

Anticancer agents and radiotherapy are ineffective for the treatment of rib chondrosarcoma. The effective treatment strategies are early diagnosis and radical surgical resection with wide and microscopically negative margins during initial surgery [5]. The methods to evaluate resection margins during surgical resection were developed by the Bone and Soft Tissue Tumor Committee of the Japanese Orthopaedic Association. Resection margins are classified into curative, wide, marginal, and intralesional margins, according to the distance from the reactive zone around a tumor. Regarding the extent of the wide resection margin, the survival rate is significantly higher with a wide resection margin of approximately 2-4 cm [6]. Evans et al. histologically classified chondrosarcoma malignancy into grades 1-3 based on pathological findings and reported that the survival rate decreases for higher grades [5]. Roos et al. reported that postoperative outcomes are poor for grade 3 chondrosarcoma exceeding 5 cm with positive resection margins [7]. Marulli et al. reported that wide surgical margins and grade 1 tumors were associated with a better prognosis and a lower recurrence rate [8]. In addition, the five-year survival rate for radical resection is reported to be 78% versus 15% for incomplete resection. They also report five-year survival rates of 97%, 57%, and 39% for grades 1, 2, and 3, respectively [8].

This patient had a grossly negative resection margin and an R1 resection (i.e., a costochondrosarcoma at the marginal margin), and the resection margin was microscopically histologically grade 1. Although no additional resection was performed in this case as the patient wished, such cases often require discussion about the significance of additional resection and the possibility of local or distant recurrence. Rib chondrosarcoma has been reported to have a relatively better outcome than general chondrosarcoma, with a five-year mortality rate of 10%, a local recurrence rate of 17%, and a metastatic rate of 12% [9]. Many prognostic factors that worsen the overall survival have been reported, including tumor diameter greater than 5 cm, positive surgical margins, and higher grade [9-11]. Local recurrence is also a poor prognostic factor, although it has been reported that negative surgical margins in the treatment of the first local recurrence were associated with a decreased risk of a second local recurrence. This is important in terms of survival for some patients who may die from local rather than distant metastases [10]. The development of distant metastases in the lungs and other organs, which are naturally more common, is also a sign of poor prognosis [12]. Current guidelines recommend extensive resection of grade II or III chondrosarcomas, but there are no specific recommendations regarding the width of the surgical margins, and there is currently no precise definition of negative margins. Generally, a resection margin of 2 cm or more is recommended, as mentioned above; however, some studies report that even 1 mm or more is acceptable [13]. However, careful long-term follow-up is essential, as studies have shown that 13% of grade 1 chondrosarcomas develop local recurrence and 1/3 of patients with local recurrence develop metastases [9]. There have been no reports of treatment decisions based on the grade of the resection margin in cases with marginal margins such as the present case, and this point of view may become important in the future. This case suggests that, when gross margins are negative and the margins are marginal, careful follow-up is possible without additional resection, depending on the histological grade of the resection margins. However, it is important to accumulate a large number of cases.

The article "Primary Chondrosarcoma of the Right Fourth Rib Resected at the Marginal Margin: A Case Report" was published in 2023. Journal: Cureus.

In cases of high-grade tumors with positive resection margins, adjuvant therapy with anticancer agents (doxorubicin), radiotherapy, and immune checkpoint inhibitors are also considered [14]. However, no clear views have been established on the effects of adjuvant therapy. It is, therefore, important to conduct clinical studies and to accumulate cases in the future.

In this case, the patient was treated with chest wall reconstruction, and careful attention to infection control is necessary if the chest wall resection is extensive. Resection with a wide margin, as in our case, may cause a flail chest, abnormal respiratory movement, or organ injury [15]. Weyant et al. recommended chest wall reconstruction when at least three ribs are resected [16]. Regarding mesh to be used, it is considered better to use mesh that keeps the thoracic cavity airtight, has high tissue affinity, is easy to handle in surgery, and is appropriately durable and elastic [14,17]. The most commonly used meshes are the Marlex mesh and expanded polytetrafluoroethylene (ePTFE) mesh. Although the ePTFE mesh has been often used in terms of antibacterial properties in recent years, it has been reported that this selection is not associated with significant differences in postoperative outcomes or recurrence of complications [18]. In addition, latissimus dorsi, pectoralis major, and rectus abdominis muscles are often used when a resection margin is wide in soft tissues. Chest wall reconstruction using synthetic polypropylene mesh and local muscle flaps is a safe and effective procedure for a chest wall defect [1].

We prefer a soft mesh that is easy to shape, lightweight, and knitted in a way to be durable. Because the soft mesh has large gaps, it also has the advantage of alleviating postoperative discomfort. In our case, three ribs were resected, and reconstruction was performed only with soft mesh without pectoralis major or latissimus dorsi muscle flaps [19]. After surgery, complications, such as incision infection and necrosis, did not occur. In addition, almost no discomfort was noted at the reconstruction site, and there was no functional problem.

## Conclusions

In this case, although the gross resection margins were negative, the R1 resection, i.e., costochondrosarcoma at the marginal margin, may be followed carefully without additional resection, depending on the histological grade of the resection margins. In cases of extensive chest wall resection, chest wall reconstruction may be useful with careful attention to infection control.
